The article "Searching Far and Genome-Wide: The Relevance of Association Studies in Amyotrophic Lateral Sclerosis" was published in 2021. Journal: Front Neurosci.

# Searching Far and Genome-Wide: The Relevance of Association Studies in Amyotrophic Lateral Sclerosis

**DOI:** 10.3389/fnins.2020.603023

**Published:** 2021-01-14

**Authors:** Kelly A. Rich, Jennifer Roggenbuck, Stephen J. Kolb

**Affiliations:** ^1^Department of Neurology, The Ohio State University Wexner Medical Center, Columbus, OH, United States; ^2^Department of Biological Chemistry and Pharmacology, The Ohio State University Wexner Medical Center, Columbus, OH, United States

**Keywords:** amyotrophic lateral sclerosis, genetic testing, gene therapy, genome, genetic variants, rare variant association study (RVAS), genome wide association studies (GWAS)

## Abstract

Genome-wide association studies (GWAS) and rare variant association studies (RVAS) are applied across many areas of complex disease to analyze variation in whole genomes of thousands of unrelated patients. These approaches are able to identify variants and/or biological pathways which are associated with disease status and, in contrast to traditional linkage studies or candidate gene approaches, do so without requiring multigenerational affected families, prior hypotheses, or known genes of interest. However, the novel associations identified by these methods typically have lower effect sizes than those found in classical family studies. In the motor neuron disease amyotrophic lateral sclerosis (ALS), GWAS, and RVAS have been used to identify multiple disease-associated genes but have not yet resulted in novel therapeutic interventions. There is significant urgency within the ALS community to identify additional genetic markers of disease to uncover novel biological mechanisms, stratify genetic subgroups of disease, and drive drug development. Given the widespread and increasing application of genetic association studies of complex disease, it is important to recognize the strengths and limitations of these approaches. Here, we review ALS gene discovery via GWAS and RVAS.

## Introduction

In the timeline of gene discovery for hereditary disease, high penetrance genes are historically identified by linkage analysis in multi-generational family studies and subsequently replicated in high-risk case-control studies of independent disease cohorts. These Mendelian genes, with highly significant (or moderately significant) effect sizes, generally represent the “low-hanging fruit” of gene discovery. Identifying the genetic underpinnings of complex diseases requires an approach to assess variation in many genes simultaneously. Genome-wide association studies (GWAS) were developed using single nucleotide variant (SNV) array technology to identify disease-associated variation in large cohorts of cases and controls and became widely adopted in the late 2000s. GWAS are able to interrogate millions of common genetic variants [minor allele frequency (MAF) > 5%] in thousands of unrelated individuals to identify associations with disease that potentially explain some percentage of disease heritability within a population (Tam et al., 2019).

Despite the impact of GWAS in identifying disease-associated genetic changes, the majority of genetic contribution to many complex diseases remains unexplained. Rare variant association studies (RVAS) extend the genome-wide approach by using massively parallel sequencing to identify less-common variants (MAF < 0.5 or 0.1%) that would be missed by GWAS (Lee et al., 2014). This has been made possible by increasing sample sizes in disease cohorts as well as advances in sequencing technology, leading to greater genomic resolution. Next generation sequencing approaches such as whole exome sequencing (WES) and whole genome sequencing (WGS), sequence the coding regions and the entirety of the genome, respectively, allowing for inclusion of rare variants into large association studies of complex disease (Kosmicki et al., 2016).

Rare variant studies extend the reach of traditional association studies by identifying rare and potentially more clinically significant variants using powerful sequencing technologies. Variants identified via GWAS only explain a fraction of missing heritability in most diseases, limiting the clinical relevance of GWAS findings (Manolio et al., 2009). Targeted candidate gene studies have revealed that rare coding variants may produce large effect sizes in complex disease, motivating further investigation into rare variant contribution (Kosmicki et al., 2016). Rare variants are known to play important roles in human disease (Rivas et al., 2011; Gudmundsson et al., 2012) and explain phenotypic differences across the disease spectrum (Cohen, 2004; Cohen et al., 2005).

While GWAS can be performed on WGS or WES, it is most commonly conducted using SNV array to maximize sample size. The associations evaluated via GWAS often do not include variants of less than 0.1% allele frequency. High-depth WGS offers the greatest opportunity for assessing low-frequency or rare variants using an RVAS approach. RVAS is able to assess both single-variants or the cumulative effects of multiple variants on a gene or region (Lee et al., 2014). The latter includes approaches such as burden tests, variance-component tests, and exponential-combination tests (Lee et al., 2014). Further, RVAS can also be used to confirm candidate associations identified via GWAS or screen a known disease-associated gene in a separate cohort (Auer and Lettre, 2015).

The typical association study includes four components; (1) accrual of a large group of individuals with the disease of interest as well as a carefully matched control group for comparison; (2) genotyping of hundreds of thousands to millions of variants in disease and control groups, traditionally via SNV arrays in GWAS and sequencing in RVAS; (3) statistical analyses to test for common- or rare-variant association with disease; and (4) prioritizing and replicating significant findings in a non-overlapping, independent cohort or performing functional experiments to examine variant consequences (Pearson, 2008). Data from association studies can be easily visualized via a Manhattan plot in which significant regions or variants appear as “skyscrapers,” an example of which is provided in Figure 1.

**FIGURE 1:** In this example Manhattan plot, each dot represents a single SNV assessed in every individual in the cohort. Genomic coordinates are displayed in ascending fashion on the *X*-axis, beginning with chromosome 1 on the left. The negative logarithm of the association p-value for each SNV is shown on the *Y*-axis. The SNVs with the strongest association will have the most negative p-value, so the negative logarithm will be greatest for these SNVs. In this example plot, SNV1 and SNV2 exceed the threshold of significance (*p* = 10^– 8^) while SNV3 does not.

As opposed to candidate gene studies assessing variation in specific genes, neither approach requires prior hypotheses of associations between genetic variants and disease. Given the widespread and increasing application of GWAS and RVAS to uncover genetic associations in complex diseases, it is important to recognize the strengths and limitations of each approach. Here we will consider the contribution of association studies in unraveling the genetic etiologies of the motor neuron disease amyotrophic lateral sclerosis (ALS).

## Strengths and Successes in Association Studies

Association studies have been used to identify significant risk loci in conditions such as type 2 diabetes (Zhao et al., 2017), schizophrenia (Li et al., 2017), hypocholesterolemia (Cohen, 2004; Cohen et al., 2005) and coronary artery disease (Nikpay et al., 2015). Beyond identifying novel disease associations, GWAS and RVAS may also serve as a first step in uncovering biological mechanisms and/or pathways for therapeutic intervention. In schizophrenia, GWAS identified a significant association signal within the major histocompatibility complex (Schizophrenia Working Group of the Psychiatric Genomics Consortium, 2014) and sparked investigation into complement factor haplotypes including C4 (Sekar et al., 2016). C4 is a known marker of synaptic pruning which was later found to be overexpressed in the brain tissue of individuals with schizophrenia. This biological context supports the theory of excessive synaptic elimination (“pruning”) as a mechanism of disease. Similarly, a GWAS approach to type 2 diabetes identified the risk locus *SLC30A8*, and follow-up investigation discovered that loss-of-function variants at this locus are protective against disease. This discovery led to the development of several drugs which aim to antagonize the product of *SLC30A8*, a zinc transporter in pancreatic islet cells (Flannick and Florez, 2016). RVAS identified rare variants in *PCSK9* as a key component of low-density lipoprotein metabolism and individuals with loss-of-function variants in this gene had consistently low cholesterol levels throughout their lifetimes (Cohen et al., 2005). Since then, three PCSK9 inhibitors have been tested in human trials, two approved in the United States (Shapiro et al., 2018). This association finding is among the most compelling examples of translation from genetic findings to therapeutic intervention.

Association studies may also provide an avenue for disease subgroup stratification, where a subgroup may have a particular clinical course (Ridker et al., 2008; Reiner et al., 2009; Owen et al., 2010; Thanabalasingham et al., 2011) or may be more likely to benefit from a certain intervention (Nelson et al., 2015). These approaches can provide insight into the impact of geoancestry in disease (Choquet et al., 2013; Wen et al., 2014; Liu et al., 2015; Minster et al., 2016; Visscher et al., 2017). GWAS and RVAS may uncover modifier genes and shed light on the contribution of multiple variants (Pigeyre et al., 2016; Whitacre et al., 2017; Tam et al., 2019). Polygenic risk scores (PRS), which predict an individual’s risk for disease based on the combination of multiple risk alleles, can be calculated using tens of thousands of association “hits” together (Wray et al., 2007). Individuals in the top 1–5% of risk profile may face a disease risk that approaches that of individuals who inherit a single monogenic pathogenic mutation (Khera et al., 2018). Informed by association results, PRS have shown modest but reliable prediction capability in a number of disease areas (Barrett et al., 2009; Schizophrenia Working Group of the Psychiatric Genomics Consortium, 2014; Hoffmann et al., 2017; Seibert et al., 2018) as well as the ability to modify risk prediction for monogenic variants (Fahed et al., 2020).

## Limitations of Association Studies

Association studies require large datasets and a stringent threshold for significance to avoid false positives. Given the nature of studying rare variants, even larger sample sizes are required with RVAS so that patients with such rare variants will be included. For less-common diseases such as ALS, the sample size required to identify risk variants of low effect size may not be feasible. Further, the overwhelming majority of association studies have been performed in European cohorts (Haga, 2010; Duncan et al., 2019). Since variant frequencies as well as linkage disequilibrium vary between ethnic groups, findings may not be applicable across racial and ethnic groups (Need and Goldstein, 2009; Gravel et al., 2011).

Perhaps most importantly, association studies, by their nature, only measure the association of a risk loci with a disease but cannot determine the impact of a SNV on lifetime risk nor the mechanism by which it confers such risk (Altshuler et al., 2008). Specifically, GWAS findings often highlight non-coding SNVs in linkage disequilibrium with several other genes or regions, making it difficult to specifically identify causal genes. Variants that are associated with disease may in fact act as direct drivers of disease progression, or such a link to disease or phenotype may not be understood, potentially because the true causal variant at that locus has not yet been identified or multiple variants at a locus must work together. Even though association to a particular variant may be statistically significant with cases compared to controls, causality cannot necessarily be assigned by the GWAS approach. Thus, GWAS may reveal synthetic associations (Dickson et al., 2010). Typical GWAS reveal multiple variants associated with disease due to linkage disequilibrium, and functional studies are necessary to determine which are truly meaningful in the context of disease (Pearson, 2008).

Additionally, in such large cohorts the cost of uniform, deep sequencing approaches such as WGS can be a prohibiting factor, so other testing approaches may be considered, each with important caveats. A number of statistical methods have been developed to increase the power of RVAS in the context of sample size limitations.

## Gene Discovery in Amyotrophic Lateral Sclerosis

Amyotrophic lateral sclerosis is a progressive neurodegenerative disorder affecting 1–2 per 100,000, involving selective loss of upper and lower motor neurons and typically resulting in death in 2–5 years (van Es et al., 2017). The discovery of multiple genes associated with ALS has led to an era of targeted gene therapies and multiple lines of mechanistic inquiry. As such, the story of gene discovery in ALS provides a useful context in which to understand the significance of GWAS- and RVAS-identified variants in a genetically heterogeneous disease population.

The first gene identified to cause familial ALS (fALS, defined as having a history of ALS in a first-, second- or third-degree relative), *SOD1*, was identified via linkage studies in 1993 (Rosen, 1993). Since then, variants in over 50 genes have been identified in individuals with both familial and sporadic ALS (an up-to-date list of these genes can be found at alsod.ac.uk). Many of these genes were identified via linkage analysis in high-penetrance fALS families and confirmed in follow-up case-control studies that utilized either Sanger sequencing, SNV arrays, or exome sequencing (Siddique et al., 1989; Hosler et al., 1998; Nishimura, 2004). Other studies utilized prior biological knowledge to identify candidate genes and then conducted case-control sequencing studies (Kwiatkowski et al., 2009; Fecto, 2011). Currently, a monogenic etiology can be identified in up to two-thirds of fALS and 10% of sporadic ALS (sALS) cases (Chia et al., 2018). As with other genetically complex diseases, traditional linkage or candidate gene approaches were responsible for the discovery of the most highly penetrant ALS genes, including *C9orf72* (DeJesus-Hernandez et al., 2011; Renton et al., 2011), *SOD1* (Rosen, 1993), and *FUS* (Kwiatkowski et al., 2009).

## Association Studies in Amyotrophic Lateral Sclerosis: Discovery and Reproducibility

The primary goal of most association studies in ALS is to identify new ALS-associated genes, either common (via GWAS) or rare (via RVAS), and this has been successful in recent years as evidenced by the identification of multiple disease-associated ALS genes (summarized in Table 1).

**TABLE 1:** A chronological overview of ALS-related genes initially identified via association studies.

**Gene(s) Identified**	**Study Type**	**Sequencing Method**	**Discovery Cohort**	**Replication Cohort**	**Reported functional validation**	**Biological role of gene product**	**Gene(s) Replicated**
*FLJ10986* (Dunckley et al., 2007)	GWAS	SNV array	386 sALS patients and 542 controls (Caucasian)	+	Western blot expression of FLJ10986 was detected in spinal cord samples from both sALS cases and controls.	Uncharacterized at time of publication. Subsequently found to be involved in carbohydrate phosphorylation (Singh et al., 2017).	
*ITPR2* (van Es et al., 2007)	GWAS	SNV array	461 ALS patients and 450 controls (Netherlands)	+ (Netherlands, Belgium, Sweden)	ITPR2 mRNA expression was greater in the peripheral blood of 126 ALS patients than in that of 126 healthy controls (p = 0.00016).	Glutamate-mediated neurotransmission, intracellular calcium concentration and apoptosis specifically in motor neurons (Gambardella et al., 2020).	
*DPP6* (van Es et al., 2008)	GWAS	SNV array	1,767 ALS patients and 1,916 controls (Netherlands, United States)	+ (Netherlands, Belgium, Sweden)		Neuronal excitability via binding of voltage-gated potassium channels. Mice with *DPP6* knockout demonstrate neuronal hyperexcitability and behavioral alterations (Lin et al., 2018).	
*UNC13A MOBKL2B* (van Es et al., 2009b)	GWAS	SNV array	2,323 sALS patients and 9,013 controls (Netherlands, United States, Ireland, Sweden Belgium)	+ (Netherlands, United States, United Kingdom, France, Ireland Poland, Germany)		*UNC13A*: Release, of neurotransmitters, such as glutamate, at neuromuscular synapses (Varoqueaux et al., 2005). *MOBKL2B*: Kinase activity (Hergovich, 2011)	
*KIFAP3* (Landers et al., 2009)	GWAS	SNV array	1,821 sALS cases and 2,258 controls (United States, Britain, France, Netherlands)	+ (United States, Europe)		*KIFAP3*: Encodes a kinesin-associated protein (Shimizu et al., 1996) Neurite outgrowth and cortical development (Ozeki et al., 2003)	
*CYP27A1* (Diekstra et al., 2012)	GWAS with eQTL	SNV array and mRNA expression	Genotyping: 2,261 sALS patients and 8,328 controls (Netherlands, Belgium, France, Ireland, United Kingdom, Sweden, United States) eQTL: 162 sALS patients and 207 controls	+		Cholesterol metabolism. Variants in this gene have been found in individuals with cerebrotendinous xanthomatosis (CTX) (Gallus et al., 2006). The progressive upper motor neuron symptoms involved in CTX overlap with those found in ALS.	*UNC13A*
*ZNF512B* (Iida et al., 2011)	GWAS	SNV array	92 ALS patients and 233 control (Japan)	+ (Japan)	ZNF512B overexpression increased TGF-β signaling and knockdown decreased TGF-β signaling. ZNF512B expression was increased in the spinal cord anterior horn motor neurons of patients.		
*CAMK1G CABIN1-SUSD2* (Deng et al., 2013)	GWAS	SNV array	506 sALS patients and 1,859 controls (Han Chinese)	+ (Han Chinese)		*CAMK1G*: Calcium kinase signaling (Takemoto-Kimura et al., 2003) *CABIN1*: Inhibition of calcineurin-mediated signal transduction (Sun et al., 1998) *SUSD2*: Cell membrane signaling (Watson et al., 2013)	
*SARM1* (Fogh et al., 2014)	GWAS	SNV array	6,100 sALS patients and 7,125 controls (Italy Netherlands, Belgium, Sweden, France, Ireland, United States, Britain)	+ (Italy, Netherlands, Germany)		Axonal degeneration (Osterloh et al., 2012)	*C9orf72*
*TBK1 NEK1* (Cirulli et al., 2015)	GWAS	Exome sequencing	2,869 patients with ALS and 6,405 controls (Caucasian)	+ (Caucasian)		*TBK1*: Autophagy (Duan et al., 2019) *NEK1*: Kinase linked to multiple cellular processes including cell cycle control and cilia repair (Thiel et al., 2011)	SOD1, TARDBP, OPTN, VCP*
*TUBA4A* (Smith et al., 2014)	RVAS	Exome sequencing	363 unrelated fALS probands and 4,331 (European American)	+ (European American)	Mutant TUB4A constructs transfected in HEK293 and primary motor neurons show altered incorporation into microtubules as well as altered microtubule polymerization and stability.	Cytoskeletal organization and maintenance (Smith et al., 2014)	MATR3**
*C21orf2 MOBP SCFD1* (van Rheenen et al., 2016)	GWAS RVAS	Genome sequencing and SNV array	1,861 ALS patients and matched controls (Australia, Belgium, France, Germany, Ireland, Italy, Netherlands and Turkey)	+ (Australia, Belgium, France, Germany, Ireland, Italy, Netherlands and Turkey)		*C21orf2:* Development and maintenance of cilia, DNA repair mechanisms (Khan et al., 2015; Wang et al., 2016). *MOBP:* Expressed in myelin, neurodegeneration (Yamamoto et al., 1994) *SCFD1:*Intracellular transport (Laufman et al., 2009)	*UNC13A, SARM1, C9orf72, TBK1, C21orf2*
*GPX3-TNIP1* (Benyamin et al., 2017)	GWAS	SNV array	13,811 sALS patients and 26,325 controls (European and Chinese)	+ (Australian)	Investigation of differential expression of GPX3 and TNIP1 between ALS patients and controls was not conclusive	*GPX3*: Antioxidant molecule functionally related to SOD1 (Chi et al., 2007) *TNIP1*: Previously associated with inflammation and immune disorders (Gateva et al., 2009; Nair et al., 2009)	*C9orf72, MOPB, SARM1, UNC13A, SCFD1*
*KIF5A* (Nicolas et al., 2018)	GWAS RVAS	SNV array (GWAS) Exome sequencing (RVAS)	20,806 ALS patients and 59,804 control samples (Caucasian European and United States)	+ (Caucasian European and United States)	Splice site prediction software (ASSEDA) predicted all *KIF5A* variants to result in aberrant splicing leading to skipping of *KIF5A* exon 27	Axonal transport (Kanai et al., 2004)	*C9orf72, TBK1, UNC13A, C21orf2, TNIP1*

sALS, sporadic ALS; fALS, familial ALS; SNV, single nucleotide variant. *This study did not assess repeat disorders including those found in *C9orf72*. **This study excluded patients with variants in several known ALS genes.

Rare variation appears to play an important role in explaining missing heritability within ALS (van Rheenen et al., 2016). As such, the field has made significant strides in applying RVAS using large, international collaborations (Smith et al., 2014; van Rheenen et al., 2016; Nicolas et al., 2018), the most recent of which identified *KIF5A* as a Mendelian ALS gene (Nicolas et al., 2018). Some GWAS studies (using SNV genotyping data) have performed RVAS (using sequencing data on smaller cohorts) as a follow-on validation step. Other approaches leverage additional sources of genetic data, such as gene expression data, to prioritize GWAS findings (Diekstra et al., 2012).

Association studies may be used to confirm previously identified findings, resulting either from early linkage studies or from other association studies in separate human ALS cohorts (Table 1). For example, *SOD1* was originally identified via linkage (Rosen, 1993) and in subsequent GWAS a clear signal was found at the *SOD1* locus (Laaksovirta et al., 2010). Additionally, association studies can help to more completely characterize a linkage finding. A 9p21.2 locus causing dominant ALS was originally discovered via linkage analysis, with multiple reports defining a minimum linkage region of 3.7 Mb including only five known genes (Luty et al., 2008; Le Ber et al., 2009; Boxer et al., 2011). This region was ultimately pinpointed to *C9orf72* in part by association studies which condensed the locus to a few genes (van Es et al., 2009b; Laaksovirta et al., 2010; Shatunov et al., 2010), providing avenues for targeted repeat-mapping in *C9orf72* (DeJesus-Hernandez et al., 2011).

Positive replication studies add support that the original finding was in fact a true association. If the replication cohort differs in geographical origin and/or phenotypic features to the original cohort, the findings may be more applicable in additional disease populations. Cross-ethnic analyses have uncovered such genes (Benyamin et al., 2017). Identifying genes and variants that are robustly replicated over time and across populations is a critical first step in characterizing the biological mechanisms underlying ALS. For example, association studies in ALS have replicated *C9orf72* as a disease-associated gene across ethnic groups (Laaksovirta et al., 2010; Shatunov et al., 2010). Additional examples of gene replication exist in small cohorts (Cronin et al., 2007; Li et al., 2009) and in larger meta-analyses (van Rheenen et al., 2016; Benyamin et al., 2017). In addition, RVAS studies have also lent support to prior GWAS findings (Kenna et al., 2016).

Nevertheless, across the board, many gene-specific replication studies have failed to replicate association findings (Chiò et al., 2009; Cronin et al., 2009; van Es et al., 2009a; Daoud et al., 2010; Fernández-Santiago et al., 2011; Fogh et al., 2011; Chen et al., 2012; Cai et al., 2014). Lack of reproducibility of association findings is common and may reflect several issues common in human genetic studies. As the risk variants often confer very small increases in risk, small sample sizes of less than 10,000 individuals are frequently underpowered to detect these risk variants. Larger study sizes (>50,000), which are most commonly assembled via large, international collaborations, are much more likely to reproduce association findings (Feliciano et al., 2018; Nishino et al., 2018; Zhang et al., 2020). The sample sizes in ALS, GWAS, and RVAS have grown steadily over time but are much smaller than those in other disease areas (Michailidou et al., 2017). Inherent population stratification also influences varying allele frequencies between individuals from different geographical regions and/or different ancestral backgrounds (Tam et al., 2019). Thus, positive associations may not be found in a subsequent study if population differences exist. Selection criteria for each cohort are not always consistent and may be subject to bias based on clinical or demographic standards (McClellan and King, 2010). Phenotypic variation in different cohorts may influence diagnosis and inclusion in genomic studies. Finally, variation in genetic testing technology and analysis as well as genotyping errors may occur between cohorts.

Genetically homogenous ethnic populations are typically selected for GWAS and RVAS because they introduce the least amount of genetic diversity and maximize the chances of identifying variants that are disease-related rather than geoancestry-related. However, the results from such cohorts are often not replicable in subsequent analyses and/or generalizable in other populations, often due to varying allele prevalence and unequal representation of different populations in case and control groups. For decades, Caucasian individuals have made up the vast majority of people studied in association studies across all diseases, including ALS (Popejoy and Fullerton, 2016). In ALS association studies, there is notable lack of replication between Asian and European ALS cohorts, which may reflect inherent population differences in SNV frequencies and disease phenotypes (Gravel et al., 2011). For example, ALS onset occurs at a younger age in Han Chinese patients and is more likely to present with bulbar-onset, as compared to limb-onset (Deng et al., 2013).

## GWAS and RVAS Studies Result in Appreciation of Relevant Mechanistic Pathways

Experiments to determine the functional consequences of ALS-associated variants in genes identified via GWAS and RVAS have further characterized the pathology underlying disease either via a specific gene product itself or the network or pathway in which it operates. Such ALS genes play roles in glutamate-mediated neurotransmission and excitability (*ITPR2* and *UNC13A*; Varoqueaux et al., 2005; Gambardella et al., 2020), regulation of neuronal excitability (*DPP6;* Lin et al., 2018), autophagy (*TBK1;* Duan et al., 2019), cytoskeletal organization (*TUBA4A;* Smith et al., 2014), and axonal transport (*KIF5A*; Nicolas et al., 2018).

Some association findings have led to promising results in *in vitro* and *in vivo* models of ALS. For example, conditional knockout of *TBK1* was reported to result in motor and cognitive defects in mice as well as pathological features typical of autophagy dysfunction (Duan et al., 2019). In SOD1^*G*93*A*^-transfected cells, *TBK1* overexpression reduced the number and size of SOD1 aggregates. *SOD1^*G*93*A*^* transgenic mice demonstrating an ALS phenotype show increased survival and decreased protein aggregates after intracerebroventricular injection of AAV vectors encoding *TBK1* (Duan et al., 2019). *TBK1* expression may have the therapeutic potential to promote autophagy even in the absence of *TBK1* variants.

Other disease pathway studies for GWAS- and RVAS-identified genes have lent support to the approaches of current therapeutic options for ALS. For example, UNC13A functions to regulate the release of neurotransmitters, such as glutamate at neuromuscular synapses (Rossner et al., 2004; Engel et al., 2016). In mice, UNC13A acts in synaptic vesicle priming, and mice lacking UNC13A demonstrate altered glutamatergic neurotransmission (Varoqueaux et al., 2005; Gambardella et al., 2020). *UNC13A* variants may therefore promote disease via glutamate-mediated excitotoxicity. Riluzole, one of two FDA-approved treatments for ALS, is a glutamate release inhibitor and can lead to a 2-3 month increase in survival for some patients (Bellingham, 2011; Dharmadasa and Kiernan, 2018). However, in clinical trials, other treatments aimed at decreasing glutamate neurotransmission have demonstrated limited or negative results (Bedlack, 2019).

## Current Impact of GWAS and RVAS on Preclinical and Clinical Therapy

Efforts to translate genetic discoveries into therapeutic clinical trials in ALS have thus far been et with limited success, in contrast to other diseases in which GWAS had led to new drugs currently in clinical trials or clinical practice (Visscher et al., 2017). The high degree of clinical and genetic heterogeneity, unknown influence of endogenous and exogenous factors on disease susceptibility, and unknown reasons for selective vulnerability of certain cell types present significant challenges to therapeutic development (Katyal and Govindarajan, 2017).

Gene-targeted clinical trials for ALS patients with variants in three genes (*FUS, C9orf72*, and *SOD1*) are underway. Antisense oligonucleotides targeted at C9orf72 mutant transcripts have shown promising results in ALS models and are currently in development for patients with *C9orf72*-related ALS (Riboldi et al., 2014; Martier et al., 2019). Recently, two approaches to down-regulate SOD1 expression in patients with SOD1-ALS [one utilizing an antisense oligonucleotide (Miller et al., 2020) and the other an adeno-associated viral vector (Mueller et al., 2020)] have been reported. The genes targeted in ALS genomic therapies were each originally identified in high-penetrance families demonstrating Mendelian inheritance, not via GWAS or RVAS. They also represent the most common, known genetic causes of ALS and were discovered prior to the widespread application of association-based technology.

There is potential utility of association studies in identifying subgroups of medication responders. This has been demonstrated in a survival analysis of patients with a particular *UNC13A* genotype who were treated with lithium carbonate (van Eijk et al., 2017). *UNC13A* was originally identified via an association study (van Es et al., 2009b). This finding suggests that GWAS and RVAS may lead to more targeted studies in the future and/or improved interpretation of clinical trial results.

Currently, results from ALS association studies are used broadly in several ways, such as improving understanding of the genetic architecture of ALS, illuminating tissue- or cell-specific pathways involving ALS-associated genes, and informing variable expressivity and penetrance of disease. Moving forward, GWAS and RVAS findings may assist in the design of combinatorial therapies that target multiple gene products and disease pathways, reflecting the proposed oligogenic nature of disease (Nguyen et al., 2018). Finally, larger, more powerful association studies may one day enable the calculation of clinical PRS to identify healthy individuals at highest risk of disease, who may be candidates for neuroprotective interventions.

## Discussion

Advances in genetic testing and identification of genetic subtypes of disease have been the cornerstone of ALS research in recent years, marked by widespread genetic testing in larger and more diverse cohorts, bioinformatic and molecular characterization of identified variants, and progress toward clinical trials for genetic subtypes of disease. Gene discovery has been driven by linkage analysis of families with high-penetrance genes, candidate gene approaches and more recently, association studies such as GWAS and RVAS. Association studies represent an attractive option for novel gene discovery because they do not require prior knowledge or hypotheses, compared with hypothesis-confirming sequencing studies.

Currently, there are no effective treatment options to halt progression of ALS and only two FDA-approved medications. Significant urgency exists within the ALS community to identify additional genetic markers of disease in order to uncover novel biological mechanisms, stratify genetic subgroups of disease, and drive drug development. Lower-penetrance genes and risk factors identified via association studies may serve as important components of combinatorial gene-targeted therapies in the future. Gene-targeted clinical trials are currently underway, though to date, no ALS genes initially identified via GWAS or RVAS have been developed for gene therapy approaches. In general, consideration of the potential of a GWAS or RVAS finding must be approached with measured expectations, particularly when such genes are quickly added to ALS clinical genetic testing panels. Association studies of common and rare genetic variation, when critically evaluated and contextualized properly, are a powerful tool in understanding the genetic basis of complex diseases such as ALS.

## Author Contributions

KR: background research. All authors: manuscript writing and development.

## Conflict of Interest

SK has received compensation for consulting from Biogen Idec, and AveXis. The remaining authors declare that the research was conducted in the absence of any commercial or financial relationships that could be construed as a potential conflict of interest.
